# Analysis of HBV and COVID-19 Coinfection Model with Intervention Strategies

**DOI:** 10.1155/2023/6908757

**Published:** 2023-09-29

**Authors:** Shewafera Wondimagegnhu Teklu

**Affiliations:** Department of Mathematics, Natural and Computational Science, Debre Berhan University, Debre Berhan, Ethiopia

## Abstract

Coinfection of hepatitis B virus (HBV) and COVID-19 is a common public health problem throughout some nations in the world. In this study, a mathematical model for hepatitis B virus (HBV) and COVID-19 coinfection is constructed to investigate the effect of protection and treatment mechanisms on its spread in the community. Necessary conditions of the proposed model nonnegativity and boundedness of solutions are analyzed. We calculated the model reproduction numbers and carried out the local stabilities of disease-free equilibrium points whenever the associated reproduction number is less than unity. Using the well-known Castillo-Chavez criteria, the disease-free equilibrium points are shown to be globally asymptotically stable whenever the associated reproduction number is less than unity. Sensitivity analysis proved that the most influential parameters are transmission rates. Moreover, we carried out numerical simulation and shown results: some parameters have high spreading effect on the disease transmission, single infections have great impact on the coinfection transmission, and using protections and treatments simultaneously is the most effective strategy to minimize and also to eradicate the HBV and COVID-19 coinfection spreading in the community. It is concluded that to control the transmission of both diseases in a population, efforts must be geared towards preventing incident infection with either or both diseases.

## 1. Introduction

Illnesses caused by tiny microorganisms like viruses, bacteria, fungi, and parasites are known as infectious diseases; for instance, COVID-19 and hepatitis B diseases are infectious diseases caused by viruses [1–3]. Hepatitis B caused by the hepatitis B virus (HBV) is one of the most common infectious diseases of the human liver. It is highly affecting the function of the human liver; according to the World Health Organization (WHO), it is one of the common and major health problem and causes chronic liver infection and puts people at high risk of death from cirrhosis of the liver and liver cancer [1, 3–5]. It is transmitted through blood contact, infected individuals' body fluids, and from mother to child during birth [6]. According to WHO, in 2019 estimated figure, 296 million individuals were living with chronic hepatitis B disease with 1.5 million new cases each year [7].

An infectious disease known as COVID-19 is a highly contagious respiratory infection caused by SARS-CoV-2 virus, and for the first time, its outbreak was investigated in China at the end of December 2019 [8–19]. On March 11, 2020, WHO declared it as one of the major and dangerous worldwide pandemic diseases [13, 20, 21]. Respiratory air droplets and touching materials contaminated with the virus are the transmission mechanisms [22–25]. It has been a great health and economic burden for many nations throughout the world [16, 22, 26]. Vaccine, washing hands by alcohol, apply face mask, isolation, quarantine, and applying social distance are currently control measures approved by WHO [21, 22, 24, 27].

Literatures of some scholars mentioned in references [1, 3, 14–16, 28–32] investigated that COVID-19 disease highly affected individuals already infected with either of HIV or TB or HBV or cholera. Literatures studied by some scholars mentioned in references [2, 4, 6, 8, 13, 14, 16–18, 20–22, 24–27, 29, 32–50] constructed and examined spreading and control of communicable disease ordinary differential method; similarly, scholars mentioned in [3, 28, 51–53] constructed and examined fractional derivative model of infectious diseases, and scholar mentioned in [1] constructed and examined a stochastic model of an infectious disease.

For a better understanding of the spreading of communicable diseases, the concept of mathematical modelling has a fundamental impact [16]. Different researchers have been formulated and analyzed mathematical models to suggest possible control mechanisms of infectious diseases. Tchoumi et al. [16] constructed malaria and COVID-19 coepidemic to examine the best control mechanisms. The result suggested that applying both single infection protection measures simultaneously is the best strategy. Teklu and Rao [46] analyzed a pneumonia and HIV codynamics with intervention measures. The result suggested that applying both vaccination and treatments has a major effect to minimize the coinfection transmission in the community. Hezam et al. [29] investigated coinfection of cholera and COVID-19 in Yemen with mathematical modelling approach. Their analysis examined the impacts of intervention strategy lockdown method, number of test kits, social distance, and individuals who are susceptible and can get CWTs for purification of water. Anwar et al. [27] investigated the impact of COVID-19 isolation intervention strategy on the spreading of COVID-19 infection using mathematical modelling approach. Ahmed et al. [28] constructed and examined an ABC-fractional order derivative model on HIV COVID-19 coepidemic transmission prediction. Ringa et al. [14] investigated the impacts of intervention strategies to reduce the burden of HIV and COVID-19 coepidemic transmission using mathematical modelling approach. Omame et al. [3] investigated a fractional order hepatitis B virus and COVID-19 coinfection model using the Atangana–Baleanu fractional derivative approach. The result shows that preventing incident infection with either or both diseases is the effective strategy to control the cocirculation of both infections. Din et al. [1] formulated and examined a stochastic model on the hepatitis B virus and COVID-19 coinfection to predict the effect of white noise intensities. The results show that persistence and eradication depend on intensity magnitude of the white noise as well as parameter values involved in the expansion of the disease. Teklu and Terefe [45] analyze COVID-19 and syphilis codynamics model to investigate the impacts of intervention measures on the disease transmission. Thangaraj and Easwaramoorthy [53] investigated a generalized fractal dimension-based comparison of edge detection methods in CT images for estimating the infection of COVID-19 disease.

Some epidemiological and medical studies proved that hepatitis B virus and COVID-19 coinfection is a common public health issue. The main aim of this study is to discover the most effective control strategy from intervention strategies applied in the proposed HBV and COVID-19 coinfection model. Literatures [1, 3] invested much effort in studying hepatitis B virus and COVID-19 coinfection but did not considered COVID-19 protection, COVID-19 treatment, hepatitis B virus protection, and hepatitis B virus treatment as prevention and control strategies simultaneously in a single model formulation which makes this study original and unpublished research work. Hence, we have highly motivated to undertake this study and fill the gap.

## 2. Mathematical Model Construction

In this study, we need to construct a deterministic model on the coinfection of HBV and COVID-19. Consider *N*(*t*) as a total human population in the study under consideration and divided it into eight distinct groups of individuals with their infection status as individuals who are susceptible to either of HBV or COVID-19 given by  *S*(*t*), who are protected form COVID-19 given by  *C*_*P*_(*t*), protected from HBV given by  *H*_*P*_(*t*), infected with COVID-19 given by  *C*_*I*_(*t*), infected with HBV given by *H*_*I*_(*t*), coinfected with HBV and COVID-19 given by *C*(*t*), recovered from COVID-19 given by *C*_*R*_(*t*), and treated from HBV infection given by *H*_*T*_(*t*) so that *N*(*t*) = *S*(*t*) + *C*_*P*_ (*t*) + *H*_*P*_(*t*) + *H*_*I*_(*t*) + *C*_*I*_(*t*) + *C*_*R*_(*t*) + *C*(*t*) + *H*_*T*_(*t*).

Individuals who are susceptible will acquire HBV at the force of infection

(1) $$\begin{array}{c} \lambda_{H}\left(t\right)=\frac{\sigma_{1}}{N}\left(H_{I}\left(t\right)+\rho_{1}C\left(t\right)\right), \end{array}$$

where  1 ≤ *ρ*_1_ < ∞ is the rate at which HBV infectivity increases and *σ*_1_ is the HBV spreading rate.

Individuals who are susceptible will acquire COVID-19 at the force of infection

(2) $$\begin{array}{c} \lambda_{C}\left(\text{t}\right)=\frac{\sigma_{2}}{N}\left(C_{I}\left(t\right)+\omega C\left(t\right)\right), \end{array}$$

where  1 ≤ *ω* < ∞ is the rate at which COVID-19 infectivity increases and *σ*_2_ is the COVID-19 spreading rate.

To construct the coinfection of HBV and COVID-19 model, let us assume the following: The parameters *γ*_1_, *γ*_2_ and (1 − *γ*_1_ − *γ*_2_) are portions of the human recruitment rate Γ that enters in the compartment *S*, *C*_*P*_ and *H*_*P*_, respectively. Population is homogeneously mixing, population is not constant, HBV-treated individuals do not transmit HBV, HBV is not vertically transmitted, and HBV and COVID-19 do not transmit simultaneous dually.

Using Table 1 (parameters), Table 2 (state variables), and given assumptions, the flow chart of the HBV and COVID-19 coinfection spreading dynamics is illustrated in Figure 1.

Based on Figure 1 the system of nonlinear differential equations of the HBV and COVID-19 coinfection is derived as

(3) $$\begin{array}{c} \frac{dS}{dt}=\left(1-\gamma_{1}-\gamma_{2}\right)\Gamma +\delta_{1}C_{P}+\delta_{2}H_{P}+\eta {\text{C}}_{R}-\left(\lambda_{H}+\lambda_{C}+\mu \right)S,\\ \frac{dC_{P}}{dt}=\gamma_{1}\Gamma -\left(\delta \lambda_{H}+\delta_{1}+\mu \right)C_{P},\\ \frac{dH_{P}}{dt}=\gamma_{2}\Gamma -\left(\delta_{2}+\mu +\sigma \lambda_{C}\right)H_{P},\\ \frac{dH_{I}}{dt}=\lambda_{H}S+\delta \lambda_{H}C_{R}-\left(\mu +\mu_{1}+\gamma +\phi \lambda_{C}\right)H_{I},\\ \frac{dC_{I}}{dt}=\lambda_{C}S+\sigma \lambda_{C}H_{P}-\left(\kappa +\mu +\mu_{2}+\varphi \lambda_{H}\right)C_{I},\\ \frac{dC}{dt}=\varphi \lambda_{H}C_{I}+\phi \lambda_{C}H_{I}+\rho \lambda_{C}H_{I}-\left(\mu +\mu_{3}+\theta \right)C,\\ \frac{dC_{R}}{dt}=\kappa C_{I}-\left(\mu +\eta \right)C_{R},\\ \frac{dH_{T}}{dt}=\gamma H_{I}+\theta C-\rho \lambda_{C}H_{T}-\mu H_{T}, \end{array}$$

with initial data

(4) $$\begin{array}{c} S\left(0\right)>0,\\ C_{P}\left(0\right)\geq 0,\\ H_{P}\left(0\right)\geq 0,\\ H_{I}\left(0\right)\geq 0,\\ C_{I}\left(0\right)\geq 0,\\ C\left(0\right)\geq 0,\\ C_{R}\left(0\right)\geq 0,\\ H_{T}\left(0\right)\geq 0. \end{array}$$

Adding all differential equations given in (3) gives

(5) $$\begin{array}{c} \frac{dN}{dt}=\Gamma -\mu N-\left(\mu_{1}H_{I}+\mu_{2}C_{I}+\mu_{3}C\right). \end{array}$$

### 2.1. Qualitative Properties of (3)

In this section, we analyzed the two basic qualitative properties of the coinfection model (3) known as the nonnegativity and boundedness of the system (3) with initial data in (4) with in the feasible region

(6) $$\begin{array}{c} \Omega =\left\{\left(S,C_{P},H_{P},H_{I},C_{I},C,C_{R},H_{T}\right)\in {\mathbb{R}}_{+}^{8},N\leq \frac{\Gamma }{\mu }\right\}. \end{array}$$

To justify the model (3) is both mathematically and biologically meaningful; it is crucial to prove that each model variable is nonnegative and bounded in the feasible region (6).

**Theorem 1 (solution nonnegativity).**

For the initial data given in (4) the model (3) solutions  *S*(*t*),  *C*_*P*_(*t*), *H*_*P*_(*t*), *H*_*I*_(*t*), *C*_*I*_(*t*),  *C*(*t*), *C*_*R*_(*t*), and *H*_*T*_(*t*) of the dynamical system (3) are nonnegative for each time *t* > 0.

**Proof**

Let  *S*(0) > 0, *C*_*P*_(0) > 0, *H*_*P*_(0) > 0, *H*_*I*_(0) > 0,  *C*_*I*_(0) > 0,  *C*(0) > 0,  *C*_*R*_(0) > 0, and *H*_*T*_(0) > 0; then for each *t* > 0, we need to show that *S* (*t*) > 0,  *C*_*P*_(*t*) > 0, *H*_*P*_(*t*) > 0,  *H*_*I*_(*t*) > 0, *C*_*I*_(*t*) > 0,  *C*(*t*) > 0,  *C*_*R*_(*t*) > 0,  and *H*_*T*_(*t*) > 0.

Define: *τ*=sup{*t* > 0 : *S* (t) > 0, *C*_*P*_(*t*) > 0, *H*_*P*_(*t*) > 0, *H*_*I*_(*t*) > 0, *C*_*I*_(*t*) > 0, *C*(*t*) > 0,*C*_*R*_(*t*) > 0 and *H*_*T*_(*t*) > 0}.

The functions  *S*(*t*), *C*_*P*_(*t*), *H*_*P*_(*t*), *H*_*I*_(*t*), *C*_*I*_(*t*), *C*(*t*), *C*_*R*_(*t*), and *H*_*I*_(*t*) are continuous so that we assured that  *τ* > 0. If *τ* = ∞, then the nonnegativity holds. But, if 0 < *τ* < ∞,  *S*(*τ*) = 0 or *C*_*P*_(*τ*) = 0 or *H*_*P*_(*τ*) = 0 or *H*_*I*_(*τ*) = 0 or *C*_*I*_(*τ*) = 0 or *C*(*τ*) = or  *C*_*R*_(*τ*) = 0 or *H*_*I*_(0) = 0.

From the first equation of the system (3) we have

(7) $$\begin{array}{c} \frac{dS}{dt}+\left(\lambda_{H}+\lambda_{C}+\mu \right)S=\left(1-\gamma_{1}-\gamma_{2}\right)\Gamma +\delta_{1}C_{P}+\delta_{2}H_{P}+\eta C_{R}, \end{array}$$

and integrating both sides, we have determined that *S*(*τ*) = *M*_1_*S*(0) + *M*_1_∫_0_^*τ*^exp^∫(*λ*_*H*_ + *λ*_*C*_ + *μ*))*dt*^((1 − *γ*_1_ − *γ*_2_)Γ + *δ*_1_*C*_*P*_(t) + *δ*_2_*H*_*P*_(t) + *ηC*_*R*_(t))*dt* > 0, where *M*_1_ = exp^−(*μτ* + ∫_0_^*τ*^(*λ*_*H*_(*w*) + *λ*_*C*_(*w*))^ > 0, *S*(0) > 0, *C*_*P*_(*t*) > 0, *H*_*P*_(*t*) > 0, *C*_*R*_(*t*) > 0, and by the definition of  *τ*, the solution  *S*(*τ*) > 0; hence, *S*(*τ*) ≠ 0.

Similarly from the second equation of system (3) we have determined that

(8) $$\begin{array}{c} \frac{dC_{P}}{dt}+\left(\delta \lambda_{H}+\delta_{1}+\mu \right)C_{P}=\gamma_{1}\Delta \;C_{P}\left(\tau \right)=M_{1}C_{P}\left(0\right)+M_{1}\int_{0}^{\tau }\exp^{\int \left(\delta_{1}+\mu +\delta \lambda_{H}\left(t\right)\right)dt}\gamma_{1}\Delta dt>0, \end{array}$$

where  *M*_1_ = exp^−(*δ*_1_*τ* + *μτ* + ∫_0_^*τ*^(*δλ*_*H*_(*w*))^ > 0, *C*_*P*_(0) > 0, and from the definition of  *τ* , we proved that *C*_*P*_(*τ*) > 0; hence, *C*_*P*_(*τ*) ≠ 0.

In the same manner, we have all the following results: *H*_*P*_(*τ*) > 0; hence,  *H*_*P*_(*τ*) ≠ 0; *H*_*I*_(*τ*) > 0; hence, *H*_*I*_(*τ*) ≠ 0; *C*_*I*_(*τ*) > 0; hence, *C*_*I*_(*τ*) ≠ 0; *C*(*τ*) > 0; hence, *C*(*τ*) ≠ 0; *C*_*R*_(*τ*) > 0; hence, *C*_*R*_(*τ*) ≠ 0; and *H*_*I*_(*τ*) > 0; hence, *H*_*I*_(*τ*) ≠ 0.

Eventually, we can conclude that *τ* = ∞, and using definition of the constant *τ*, all the model (3) solutions are nonnegative.

**Theorem 2 (model solution boundedness).**

The feasible region *Ω* stated in (6) is bounded in the space ℝ_+_^8^.

**Proof**

Using the proof of Theorem 1, equation (5) and in the absence of infections, we have determined that  *dN*/*dt* ≤ Δ − *μN*. Applying the standard comparison theorem criteria, we derived the integral ∫(*dN*/(Δ − *μN*)) ≤ ∫*dt* and the result −(1/*μ*)ln(Δ − *μN*) ≤ *t* + *k*, where *k* is an arbitrary constant. After a number of steps of computations, we have determined that the final result 0 ≤ *N* (*t*) ≤ Δ/*μ* means the dynamical system (3) solutions with initial data (4) are bounded in the region (6).

## 3. Mathematical Analysis of the Dynamical Systems

To analyze the complete dynamical system (3) we need the following basic information about the HBV and COVID-19 single infection spreading dynamics.

### 3.1. Mathematical Analysis of the HBV Submodel

The HBV submodel of the dynamical system (3) at  *C*_*P*_ = *C*_*I*_ = *C* = *C*_*R*_ = 0 is derived as

(9) $$\begin{array}{c} \frac{dS}{dt}=\left(1-\gamma_{2}\right)\Gamma +\delta_{2}H_{P}-\left(\lambda_{H}+\mu \right)S,\\ \frac{dH_{P}}{dt}=\gamma_{2}\Delta -\left(\delta_{2}+\mu \right)H_{P},\\ \frac{dH_{I}}{dt}=\lambda_{H}S-\left(\mu +\mu_{1}+\gamma \right)H_{I},\\ \frac{dH_{T}}{dt}=\gamma H_{I}-\mu H_{T}, \end{array}$$

where the total number of individuals in the HBV submodel is represented by *N*_1_(*t*) = *S*(*t*) + *H*_*P*_(*t*) + *H*_*I*_(*t*) + *H*_*T*_(*t*), with infection rate  *λ*_*H*_ = (*σ*_1_/*N*_1_)*H*_*I*_ and initial data  *S*(0) > 0,  *H*_*P*_(0) ≥ 0,  *H*_*I*_(0) ≥ 0, and  *H*_*T*_(0) ≥ 0. In $\Omega_{1}=\left\{\begin{array}{c} \left(S,H_{P},H_{I},H_{T}\right)\in {{\mathbb{R}}^{4}}_{+},N_{1}\leq \Gamma /\mu \end{array}\right\}$, it is not difficult to prove that the region *Ω*_1_ is both positive invariant and global attractor of each nonnegative solution of the HBV infection system (9). Therefore, one can consider that the dynamical system (9) is both biologically and mathematically meaningful in the region *Ω*_1_.

#### 3.1.1. Dynamical System (3) DFE Stability

The disease-free equilibrium (DFE) point of the HBV infection submodel (9) is calculated by putting every equation of (9) as zero in the absence of infections and treated groups. After some computation steps, we have determined the DFE as *E*_*H*_^0^ = (Δ/*μ*((*α*_2_ + *μ*(1 − *π*_2_))/(*α*_2_ + *μ*)), Δ*π*_2_/(*α*_2_ + *μ*), 0, 0).

Using the van den Driessche and Warmouth well-known method illustrated in [54] we can calculate the submodel (9) reproduction number and linear stability of its DFE. In a similar manner of [54] we computed the matrices

(10) $$\begin{array}{c} F=\left(\begin{array}{cc} \frac{\sigma_{1}}{N_{1}^{0}}{\text{S}}^{0} & 0\\ 0 & 0 \end{array}\right)=\left(\begin{array}{cc} \frac{\sigma_{1}\delta_{2}+\sigma_{1}\mu \left(1-\gamma_{2}\right)}{\delta_{2}+\mu } & 0\\ 0 & 0 \end{array}\right),\\ V=\left(\begin{array}{cc} \mu +\mu_{1}+\gamma & 0\\ -\gamma & \mu \end{array}\right). \end{array}$$

Finally, using the method in [54] and after some steps of computations, we have determined that the submodel (9) reproduction number as the maximum eigenvalue in magnitude of the product matrix *FV*^−1^ represented by

(11) $$\begin{array}{c} R_{H}=\frac{\sigma_{1}\left(\mu \left(1-\gamma_{2}\right)+\delta_{2}\right)}{\left(\gamma +\mu +\mu_{1}\right)\left(\mu +\delta_{2}\right)}. \end{array}$$

Because the calculated reproduction number of HBV submodel given by *ℛ*_*H*_ is defined as the average number of secondary infections caused by a single infected person during his life infectious period in a susceptible group, the submodel has a local stable DFE,  *E*_*H*_^0^ = (Γ/*μ*((*δ*_2_ + *μ*(1 − *γ*_2_))/(*δ*_2_ + *μ*)), Γ*γ*_2_/(*δ*_2_ + *μ*), 0, 0) whenever *ℛ*_*H*_ < 1 and unstable whenever *ℛ*_*H*_ > 1.

#### 3.1.2. Endemic Equilibrium Existence and Uniqueness

Making the submodel (9) equation right-hand side as zero and calculated for the nonzero solution, we derived the following results:

(12) $$\begin{array}{c} S^{*}=\frac{\left(1-\gamma_{2}\right)\Gamma \left(\delta_{2}+\mu \right)+\delta_{2}\gamma_{2}\Gamma }{\left(\delta_{2}+\mu \right)\left(\mu +\lambda_{H}^{*}\right)},\\ H_{I}^{*}=\frac{\gamma_{2}\Gamma \left(\delta_{2}+\mu \right)\lambda_{H}^{*}+\delta_{2}\gamma_{2}\Gamma \lambda_{H}^{*}}{\left(\mu +\mu_{1}+\gamma \right)\left(\delta_{2}+\mu \right)\left(\mu +\lambda_{H}^{*}\right)},\\ H_{T}^{*}=\frac{\left(1-\gamma_{2}\right)\mu \Gamma \gamma \left(\delta_{2}+\mu \right)\lambda_{H}^{*}+\delta_{2}\gamma_{2}\mu \Gamma \gamma \lambda_{H}^{*}}{\left(\mu +\mu_{1}+\gamma \right)\left(\delta_{2}+\mu \right)\left(\mu +\lambda_{H}^{*}\right)}. \end{array}$$

Let us put *m*_1_ = *δ*_2_ + *μ* and *m*_2_ = *μ* + *μ*_1_ + *γ* and substitute *H*_*I*_^∗^ in the incidence rate of HBV and calculated as

(13) $$\begin{array}{c} \lambda_{H}^{*}=\frac{\sigma_{1}\left(1-\gamma_{2}\right)\Delta m_{1}\lambda_{H}^{*}+\sigma_{1}\delta_{2}\gamma_{2}\Gamma \lambda_{H}^{*}}{\left(1-\gamma_{2}\right)\Gamma m_{1}m_{2}+\delta_{2}\gamma_{2}\Gamma m_{2}+\gamma_{2}\Gamma m_{2}\left(\mu +\lambda_{H}^{*}\right)+\left(1-\gamma_{2}\right)\Gamma m_{1}\lambda_{H}^{*}+\delta_{2}\gamma_{2}\Gamma \lambda_{H}^{*}\left(1+\mu \gamma \right)+\left(1-\gamma_{2}\right)\mu \Gamma \gamma m_{1}\lambda_{H}^{*}}, \end{array}$$

and simplifying the result, we determined the nonzero linear equation given by

(14) $$\begin{array}{c} L_{1}\lambda_{H}^{*}+L_{0}=0, \end{array}$$

where

(15) $$\begin{array}{c} L_{1}=-\gamma_{2}\Gamma m_{2}-\left(1-\gamma_{2}\right)\Gamma m_{1}-\delta_{2}\gamma_{2}\Gamma -\left(1-\gamma_{2}\right)\mu \Gamma \gamma m_{1}-\delta_{2}\gamma_{2}\mu \Gamma \gamma <0, \end{array}$$

(16) $$\begin{array}{c} L_{0}=m_{1}m_{2}\left[R_{H}-1\right]>0\text{ whenever }R_{H}>1. \end{array}$$

From equation (14) we computed for nonnegative infection rate given by the result

(17) $$\begin{array}{c} \;\lambda_{H}^{*}=\frac{-L_{0}}{L_{1}}=\frac{-m_{1}m_{2}\left[R_{H}-1\right]}{-\left[\gamma_{2}\Gamma m_{2}+\left(1-\gamma_{2}\right)\Gamma m_{1}+\delta_{2}\gamma_{2}\Gamma +\left(1-\gamma_{2}\right)\mu \Gamma \gamma m_{1}+\delta_{2}\gamma_{2}\mu \Gamma \gamma \right]}, \end{array}$$

that is,

(18) $$\begin{array}{c} \lambda_{H}^{*}=\frac{-L_{0}}{L_{1}}=\frac{m_{1}m_{2}\left[R_{H}-1\right]}{\left[\gamma_{2}\Gamma m_{2}+\left(1-\gamma_{2}\right)\Gamma m_{1}+\delta_{2}\gamma_{2}\Gamma +\left(1-\gamma_{2}\right)\mu \Gamma \gamma m_{1}+\delta_{2}\gamma_{2}\mu \Gamma \gamma \right]}>0, \end{array}$$

only if *ℛ*_*H*_ > 1.

Depending on the result *λ*_*H*_^∗^ > 0 obtained above, we can conclude that the submodel (9) has a positive unique endemic equilibrium point only whenever *ℛ*_*H*_ > 1.

**Theorem 3 .**

The dynamical system (9) has a positive unique endemic equilibrium point only whenever *ℛ*_*H*_ > 1.

#### 3.1.3. Global Asymptotic Stability of DFE

**Theorem 4 (Castillo-Chavez et al.'s stability condition explained in [34]).**

If the dynamical system (9) can be illustrated as

(19) $$\begin{array}{c} \frac{dU}{dt}=I\left(U,V\right),\\ \frac{dV}{dt}=J\left(U,V\right),J\left(U^{0},0\right)=0, \end{array}$$

where *U* ∈ ℝ^*k*^ be noninfected components and *V* ∈ ℝ^*m*^ be the infected components which includes the treated group and *E*_*H*_^0^ = (*U*^0^, 0) represents the DFE of the sum-model (9).

Let us assume the following:

- For (*dU*/*dt*) = *I*(*U*^0^, 0),  *Y*^0^ has a global asymptotic stability
- $J\left(U,V\right)=HU-\overset{ˇ}{J}\left(U,V\right)$, $\;\overset{ˇ}{J}\left(U,V\right)\geq 0$ for (*U*, *V*) ∈ *Ω*_1_, where *H* = *D*_*U*_*J*(*U*^0^, 0) is an *M*-matrix, i.e., the off diagonal elements of *H* are nonnegative and *Ω*_1_ is the region in which the system makes epidemiological sense. The DFE of the submodel (9) given by *E*_*H*_^0^ = (*U*^0^, 0) has a global asymptotic stability provided that *ℛ*_*H*_ < 1

**Theorem 5 .**

The DFE *E*_*H*_^0^ = (Γ/*μ*((*δ*_2_ + *μ*(1 − *γ*_2_))/(*δ*_2_ + *μ*)), Γ*γ*_2_/(*δ*_2_ + *μ*), 0, 0) of the HBV dynamical system (9) has a global asymptotic stability provided that  *ℛ*_*H*_ < 1 and the sufficient conditions sated by Theorem 3 are satisfied.

**Proof**

Using Theorem 4 for the HBV dynamical system (9) we have obtained the matrices represented by

(20) $$\begin{array}{c} \frac{dU}{dt}=I\left(U,V\right)=\left[\begin{array}{c} \left(1-\gamma_{2}\right)\Gamma +\delta_{2}H_{P}-\left(\lambda_{H}+\mu \right)S\\ \gamma_{2}\Gamma -\left(\delta_{2}+\mu \right)H_{P} \end{array}\right],\\ \frac{dV}{dt}=J\left(U,V\right)=\left[\begin{array}{c} \lambda_{H}\text{S}-\left(\mu +\mu_{1}+\gamma \right)H_{I}\\ \gamma H_{I}-\mu H_{T} \end{array}\right],\\ I\left(Y^{0},0\right)=\left[\begin{array}{c} \left(1-\gamma_{2}\right)\Gamma +\delta_{2}H_{P}^{0}-\mu S^{0}\\ \gamma_{2}\Gamma -\left(\delta_{2}+\mu \right)H_{P}^{0} \end{array}\right], \end{array}$$

where *U*^0^ = (*S*^0^, *H*_*P*_^0^) = (((1 − *γ*_2_)Γ(*δ*_2_ + *μ*) + *δ*_2_*γ*_2_Γ)/*μ*(*δ*_2_ + *μ*), *γ*_2_Γ/(*δ*_2_ + *μ*)) has a global stability and satisfies criteria (i) of Theorem 4 and

(21) $$\begin{array}{c} H=D_{U}J\left(U^{*},0\right)=\left[\begin{array}{cc} \sigma_{1}-\left(\mu +\mu_{1}+\gamma \right) & 0\\ \gamma & -\mu \end{array}\right]. \end{array}$$

We computed the result given by

(22) $$\begin{array}{c} \overset{ˇ}{J}\left(U,V\right)=\left[\begin{array}{c} {\overset{ˇ}{J}}_{1}\left(U,V\right)\\ {\overset{ˇ}{J}}_{2}\left(U,V\right) \end{array}\right]=\left[\begin{array}{c} \sigma_{1}H_{I}-\frac{\sigma_{1}H_{I}}{N_{1}}S\\ 0 \end{array}\right]=\left[\begin{array}{c} \sigma_{1}H_{I}\left(1-\frac{S}{N_{1}}\right)\\ 0 \end{array}\right]. \end{array}$$

Here, because *S* ≤ *N*_1_, we can prove that *S*/*N*_1_ ≤ 1 and ${\overset{ˇ}{J}}_{1}\left(U,V\right)\geq 0$ that satisfied criteria (ii) of Theorem 4, and hence, the DFE of the dynamical system (9) given by *E*_*H*_^0^ = (Γ/*μ*((*δ*_2_ + *μ*(1 − *γ*_2_))/(*δ*_2_ + *μ*)), Γ*γ*_2_/(*δ*_2_ + *μ*), 0, 0) has a global asymptotic stability whenever  *ℛ*_*H*_ < 1.

Epidemiologically, it means that the HBV single infection will die out in the community provided that  *ℛ*_*H*_ < 1 in this case the total number of population is going up.

### 3.2. The COVID-19 Subdynamical System

By making  *H*_*P*_ = *H*_*I*_ = *C* = *H*_*T*_ = 0 for the dynamical system (3) the COVID-19 subdynamical system is derived as

(23) $$\begin{array}{c} \frac{dS}{dt}=\left(1-\gamma_{1}\right)\Gamma +\delta_{1}C_{P}+\eta C_{R}-\left(\lambda_{C}+\mu \right)S,\\ \frac{dC_{P}}{dt}=\gamma_{1}\Gamma -\left(\delta_{1}+\mu \right)C_{P},\\ \frac{dC_{I}}{dt}=\lambda_{C}S-\left(\kappa +\mu +\mu_{2}\right)C_{I},\\ \frac{dC_{R}}{dt}=\kappa C_{I}-\left(\mu +\eta \right)C_{R}, \end{array}$$

with force of infection for COVID-19 only infection represented by

(24) $$\begin{array}{c} \lambda_{C}=\frac{\sigma_{2}}{N_{2}}C_{I}\left(t\right), \end{array}$$

with initial data given by  *S*(0) > 0, *C*_*P*_(0) ≥ 0, *C*_*I*_(0) ≥ 0, *C*_*R*_(0) ≥ 0 and total number of individuals given by  *N*_2_(*t*) = *S*(*t*) + *C*_*P*_(*t*) + *C*_*I*_(*t*) + *C*_*R*_(*t*).

In $\Omega_{2}=\left\{\begin{array}{c} \left(S,C_{P},C_{I},C_{R}\right)\in {{\mathbb{R}}^{4}}_{+},N_{2}\leq \Gamma /\mu \end{array}\right\}$, it is not difficult to prove that the region *Ω*_2_ is both positive invariant and global attractor of each nonnegative solution of the subdynamical system (23). Therefore, one can consider that the region *Ω*_2_ is both biologically and mathematically meaningful.

#### 3.2.1. The Subdynamical System DFE Stability

The COVID-19 subdynamical system (23) disease-free equilibrium (DFE) is calculated by making the system (23) equal to zero in the absence infection and recovery groups, i.e., *C*_*I*_^0^ = *C*_*R*_^0^ = 0, and therefore, the COVID-19 subdynamical system (23) is given as *E*_*C*_^0^ = (S^0^, *C*_*P*_^0^, *C*_*I*_^0^ *C*_*R*_^0^) = (Γ/*μ*((*δ*_1_ + *μ*(1 − *γ*_1_))/(*δ*_1_ + *μ*)), Γ*γ*_1_/(*δ*_1_ + *μ*), 0, 0).

The COVID-19 subdynamical system (23) effective reproduction is the average total number of new infection caused by a single infectious person through the community. By applying the criteria stated in [54] and the COVID-19 subdynamical system (23) effective reproduction number is calculated as  *ℛ*_*C*_ = (*σ*_2_(*μ*(1 − *γ*_1_) + *δ*_1_))/((*μ* + *μ*_2_ + *κ*)(*μ* + *δ*_1_)).

Based on the next generation matrix, the DFE point of the COVID-19 subdynamical system given by  *E*_*C*_^0^ = (S^0^, *C*_*P*_^0^, *C*_*I*_^0^ *C*_*R*_^0^) = (Γ/*μ*((*δ*_1_ + *μ*(1 − *γ*_1_))/(*δ*_1_ + *μ*)), Γ*γ*_1_/(*δ*_1_ + *μ*), 0, 0) has a local asymptotic stablty whenever *ℛ*_*C*_ < 1 and unstable whenever *ℛ*_*C*_ > 1.

#### 3.2.2. Endemic Equilibrium Existence and Uniqueness

The COVID-19 subdynamical system (23) endemic equilibrium point(s) is/are computed by setting its right-hand side equal to zero and determined as

(25) $$\begin{array}{c} S^{*}=\frac{\left(1-\gamma_{1}\right)\Gamma n_{1}n_{2}n_{3}+\delta_{1}\gamma_{1}\Gamma n_{2}n_{3}}{n_{1}n_{2}n_{3}\left(\lambda_{C}^{*}+\mu \right)-n_{1}\eta \kappa \lambda_{C}^{*}},\\ C_{P}^{*}=\frac{\gamma_{1}\Gamma }{n_{1}},\\ C_{I}^{*}=\frac{\left(1-\gamma_{1}\right)\Gamma n_{1}n_{2}n_{3}\lambda_{C}^{*}+\delta_{1}\gamma_{1}\Gamma n_{2}n_{3}\lambda_{C}^{*}}{n_{1}{n_{2}}^{2}n_{3}\left(\lambda_{C}^{*}+\mu \right)-n_{1}n_{2}\eta \kappa \lambda_{C}^{*}},\\ C_{R}^{*}=\frac{\left(1-\gamma_{1}\right)\Gamma n_{1}n_{2}n_{3}\kappa \lambda_{C}^{*}+\delta_{1}\gamma_{1}\Gamma n_{2}n_{3}\kappa \lambda_{C}^{*}}{n_{1}{n_{2}}^{2}{n_{3}}^{2}\left(\lambda_{C}^{*}+\mu \right)-n_{1}n_{2}n_{3}\eta \kappa \lambda_{C}^{*}}, \end{array}$$

where *n*_1_ = *δ*_1_ + *μ*,  *n*_2_ = *κ* + *μ* + *μ*_2_, and *n*_3_ = *μ* + *η*.

We can substitute *C*_*I*_^∗^ stated in (25) in (24) and calculated as *N*_2_^∗^*λ*_*C*_^∗^ = *σ*_2_*C*_*I*_^∗^ and gives as

(26) $$\begin{array}{c} \left(1-\gamma_{1}\right)\Gamma n_{1}{n_{2}}^{2}{n_{3}}^{2}+\delta_{1}\gamma_{1}\Gamma {n_{2}}^{2}{n_{3}}^{2}+\gamma_{1}\Gamma {n_{2}}^{2}{n_{3}}^{2}\lambda_{C}^{*}+\gamma_{1}\Gamma {n_{2}}^{2}{n_{3}}^{2}\mu +\left(1-\gamma_{1}\right)\Gamma n_{1}n_{2}{n_{3}}^{2}\lambda_{C}^{*}-\gamma_{1}\Gamma n_{2}n_{3}\eta \kappa \lambda_{C}^{*}+\delta_{1}\gamma_{1}\Gamma n_{2}{n_{3}}^{2}\lambda_{C}^{*}+\left(1-\gamma_{1}\right)\Gamma n_{1}n_{2}n_{3}\kappa \lambda_{C}^{*}+\delta_{1}\gamma_{1}\Gamma n_{2}n_{3}\kappa \lambda_{C}^{*}-\sigma_{2}\left(1-\gamma_{1}\right)\Gamma n_{1}n_{2}{n_{3}}^{2}-\sigma_{2}\delta_{1}\gamma_{1}\Gamma n_{2}{n_{3}}^{2}=0. \end{array}$$

By arranging equation (26) we determined the linear equation given by

(27) $$\begin{array}{c} B_{1}\lambda_{C}^{*}+B_{0}=0, \end{array}$$

where

(28) $$\begin{array}{c} B_{1}=\gamma_{1}\Gamma n_{2}n_{3}\left(n_{2}n_{3}-\eta \kappa \right)+\left(1-\gamma_{1}\right)\Gamma n_{1}n_{2}n_{3}\left(n_{3}+\kappa \right)+\delta_{1}\gamma_{1}\Gamma n_{2}n_{3}\left(n_{3}+\kappa \right)>0, \end{array}$$

(29) $$\begin{array}{c} B_{0}=\Gamma {n_{2}n_{3}}^{2}\left(\left(1-\gamma_{1}\right)n_{1}n_{2}+\delta_{1}\gamma_{1}n_{2}\right)\left[1-R_{C}\right]<0, \end{array}$$

whenever *ℛ*_*C*_ > 1.

Using (27) we derived the positive infection rate

(30) $$\begin{array}{c} \lambda_{C}^{*}=-\frac{B_{0}}{B_{1}}=\frac{\Gamma {n_{2}n_{3}}^{2}\left(\gamma_{2}n_{1}n_{2}+\delta_{1}\gamma_{1}n_{2}\right)\left[R_{C}-1\right]}{\gamma_{1}\Gamma n_{2}n_{3}\left(n_{2}n_{3}-\eta \kappa \right)+\gamma_{2}\Gamma n_{1}n_{2}n_{3}\left(n_{3}+\kappa \right)+\delta_{1}\gamma_{1}\Gamma n_{2}n_{3}\left(n_{3}+\kappa \right)}>0, \end{array}$$

only whenever *ℛ*_*C*_ > 1.

Hence, subdynamical system (23) has a unique nonnegative (in this case positive) endemic equilibrium point provided that *ℛ*_*C*_ > 1.

**Theorem 6 .**

The COVID-19 subdynamical system (23) has a positive and unique positive endemic equilibrium whenever *ℛ*_*C*_ > 1.

#### 3.2.3. DFE Global Asymptotic Stability

**Theorem 7 .**

The DFE point of the COVID-19 subdynamical system (23) given by *E*_*C*_^0^ = (((1 − *γ*_1_)Γ(*δ*_1_ + *μ*) + *δ*_1_*γ*_1_Γ)/(*μ*(*δ*_1_ + *μ*)), *γ*_1_Γ/(*δ*_1_ + *μ*), 0, 0) has a global asymptotic stability whenever  *ℛ*_*C*_ < 1, and the two sufficient criteria stated in Theorem 4 are qualified.

**Proof**

Now using the criteria in Theorem 4 for the COVID-19 subdynamical system (23) and letting *U* ∈ ℝ^2^ to be the noninfected components, *V* ∈ ℝ^2^ to be the infected components including the COVID-19 recovery group. Now we derived the matrices given by

(31) $$\begin{array}{c} \frac{dU}{dt}=I\left(U,V\right)=\left[\begin{array}{c} \left(1-\gamma_{1}\right)\Gamma +\delta_{1}C_{P}+\eta C_{R}-\left(\lambda_{C}+\mu \right)S\\ \gamma_{1}\Gamma -\left(\delta_{1}+\mu \right)C_{P} \end{array}\right],\\ \frac{dV}{dt}=J\left(U,V\right)=\left[\begin{array}{c} \lambda_{C}S-\left(\kappa +\mu +\mu_{2}\right)H_{I}\\ \kappa H_{I}-\left(\mu +\eta \right){\text{C}}_{R} \end{array}\right],\\ I\left(U,0\right)=\left[\begin{array}{c} \left(1-\gamma_{1}\right)\Gamma +\delta_{1}C_{P}-\mu S\\ \gamma_{1}\Gamma -\left(\delta_{1}+\mu \right)C_{P} \end{array}\right],\\ H=D_{W}J\left(U^{*},0\right)=\left[\begin{array}{cc} \frac{\sigma_{2}S^{0}}{S^{0}+C_{P}^{0}}-\left(\kappa +\mu +\mu_{2}\right) & 0\\ \kappa & -\left(\mu +\eta \right) \end{array}\right]. \end{array}$$

After a number of some steps of computations, we derived the following:

(32) $$\begin{array}{c} \overset{ˇ}{J}\left(U,V\right)=\left[\begin{array}{c} {\overset{ˇ}{J}}_{1}\left(U,V\right)\\ {\overset{ˇ}{J}}_{2}\left(U,V\right) \end{array}\right]=\begin{array}{c} \left[-\begin{array}{c} \frac{\sigma_{2}S^{0}H_{I}}{S^{0}+C_{P}^{0}}+\frac{\beta_{2}H_{I}S}{N_{2}}\\ 0 \end{array}\right] \end{array}=\left[\begin{array}{c} \sigma_{2}H_{I}\left(-\frac{S^{0}}{S^{0}+C_{P}^{0}}+\frac{S}{N_{2}}\right)\\ 0 \end{array}\right]. \end{array}$$

Because *S* ≤ *S*^0^ and *C*_*P*_ < *C*_*P*_^0^ , we can show that (*S*^0^/(*S*^0^ + *C*_*P*_^0^)*S*^0^ + *C*_*P*_^0^) ≥ (*S*/*N*_2_) and $\;{\overset{ˇ}{J}}_{1}\left(U,V\right)\geq 0;$ thus, the DFE point *E*_*C*_^0^ = (((1 − *γ*_1_)Γ(*δ*_1_ + *μ*) + *δ*_1_*γ*_1_Γ)/(*μ*(*δ*_1_ + *μ*)), *γ*_1_Γ/(*δ*_1_ + *μ*), 0, 0) of the COVID-19 subdynamical system (23) has a global asymptotic stability whenever  *ℛ*_*C*_ < 1.

Epidemiologically, it means that the COVID-19 single infection dies out whenever  *ℛ*_*C*_ < 1, and the total human population is going up [33].

### 3.3. Mathematical Analysis of HBV and COVID-19 Coinfection System

After analyzing the spreading dynamics of the HBV and COVID-19 single infection given in equation (9) and equation (23), respectively, the complete dynamical system given in (3) can be analyzed in the region *Ω* stated in (6).

#### 3.3.1. DFE Stability

The DFE of the coinfection dynamical system (3) represented by *E*_*HC*_^0^ is calculated by setting each equation of the system as zero at  *H*_*I*_ = *C*_*I*_ = *C*_*R*_ = C = *H*_*T*_ = 0, and we have determined as

(33) $$\begin{array}{c} E_{HC}^{0}=\left({\text{S}}^{0},C_{P}^{0},H_{P}^{0},H_{I}^{0},C_{I}^{0},,{\text{C}}^{0},C_{R}^{0},H_{T}^{0}\right)=\left.\frac{\left(1-\gamma_{1}-\gamma_{2}\right)\Gamma \left(\delta_{1}+\mu \right)\left(\delta_{2}+\mu \right)+\delta_{1}\gamma_{1}\Gamma +\delta_{2}\gamma_{2}\Gamma \left(\delta_{1}+\mu \right)}{\mu \left(\delta_{1}+\mu \right)\left(\delta_{2}+\mu \right)},\frac{\gamma_{1}\Gamma }{\delta_{1}+\mu },\frac{\gamma_{2}\Gamma }{\delta_{2}+\mu },0,0,0,0,0\right). \end{array}$$

In a similar manner of the single infection models analyzed above applying the criteria explained in [54], the effective reproduction of the complete model (3) denoted as  *ℛ*_*HC*_ can be computed as

(34) $$\begin{array}{c} FV^{-1}=\left[\begin{array}{ccccc} \frac{\sigma_{1}\left(\mu \left(1-\gamma_{2}\right)+\delta_{2}\right)}{\left(\gamma +\mu +\mu_{1}\right)\left(\mu +\delta_{2}\right)} & 0 & 0 & 0 & 0\\ 0 & \frac{\sigma_{2}\left(\mu \left(1-\gamma_{1}\right)+\delta_{1}\right)}{\left(\mu +\mu_{2}+\kappa \right)\left(\mu +\delta_{1}\right)} & 0 & 0 & 0\\ 0 & 0 & 0 & 0 & 0\\ 0 & 0 & 0 & 0 & 0\\ 0 & 0 & 0 & 0 & 0 \end{array}\right]. \end{array}$$

The effective reproduction number of the COVID-19 and HBV coinfected dynamical system (3) is the maximum eigenvalue in magnitude of the product matrix *F*.*V*^−1^, and it is given by *ℛ*_*HC*_^0^ = max{(*σ*_1_(*μ*(1 − *γ*_2_) + *δ*_2_))/((*γ* + *μ* + *μ*_1_)(*μ* + *δ*_2_)), (*σ*_2_(*μ*(1 − *γ*_1_) + *δ*_1_))/((*μ* + *μ*_2_ + *κ*)(*μ* + *δ*_1_))}, where *ℛ*_*HC*_^0^ = max{*ℛ*_*H*_, *ℛ*_*C*_}, *ℛ*_*H*_ to be the HBV submodel (9) effective reproduction number and  *ℛ*_*C*_ and *ℛ*_*HC*_^0^ to be the effective reproduction numbers of the COVID-19 single infection dynamical system (23) and the complete dynamical system (3), respectively.

Based on the definition of next generation matrix operator criteria in [54] the DFE point of the complete dynamical system (3) given by

(35) $$\begin{array}{c} E_{HC}^{0}=\left({\text{S}}^{0},C_{P}^{0},H_{P}^{0},H_{I}^{0},C_{I}^{0},,{\text{C}}^{0},C_{R}^{0},H_{T}^{0}\right)=\left.\frac{\left(1-\gamma_{1}-\gamma_{2}\right)\Gamma \left(\delta_{1}+\mu \right)\left(\delta_{2}+\mu \right)+\delta_{1}\gamma_{1}\Gamma +\delta_{2}\gamma_{2}\Gamma \left(\delta_{1}+\mu \right)}{\mu \left(\delta_{1}+\mu \right)\left(\delta_{2}+\mu \right)},\frac{\gamma_{1}\Gamma }{\delta_{1}+\mu },\frac{\gamma_{2}\Gamma }{\delta_{2}+\mu },0,0,0,0,0\right) \end{array}$$

has a local asymptotic stability whenever *ℛ*_*HC*_ < 1 and unstable whenever *ℛ*_*HC*_ > 1.

#### 3.3.2. The Complete Dynamical System (3) Endemic Equilibrium

The possible endemic equilibrium point of the dynamical system (3) is calculated by setting every equation equal to zero and is derived as

(36) $$\begin{array}{c} S^{*}=\frac{\left(1-\gamma_{1}-\gamma_{2}\right)\Gamma +\delta_{1}C_{P}^{*}+\delta_{2}C_{P}^{*}+\eta C_{R}^{*}}{\left(\lambda_{H}^{*}+\lambda_{C}^{*}+\mu \right)},\\ C_{P}^{*}=\frac{\gamma_{1}\Gamma }{\left(\delta \lambda_{H}^{*}+\delta_{1}+\mu \right)},\\ H_{P}^{*}=\frac{\gamma_{2}\Gamma }{\left(\delta \delta_{2}+\mu +\sigma \lambda_{C}^{*}\right)},\\ \;H_{I}^{*}=\frac{\lambda_{H}^{*}S^{*}+\delta \lambda_{H}^{*}C_{P}^{*}}{\left(\mu +\mu_{1}+\gamma +\phi \lambda_{C}^{*}\right)},\\ C_{I}^{*}=\frac{\lambda_{C}^{*}S^{*}+\delta \lambda_{C}^{*}H_{P}^{*}}{\left(\kappa +\mu +\mu_{2}+\varphi \lambda_{H}^{*}\right)},\\ C^{*}=\frac{\varphi \lambda_{H}^{*}C_{I}^{*}+\phi \lambda_{C}^{*}H_{I}^{*}+\rho \lambda_{C}^{*}H_{T}^{*}}{\left(\mu +\mu_{3}+\theta \right)},\\ C_{R}^{*}=\frac{\kappa C_{I}^{*}}{\left(\mu +\eta \right)},\\ H_{T}^{*}=\frac{\gamma \;H_{I}^{*}+\theta C^{*}}{\left(\rho \lambda_{C}^{*}+\mu \right)}. \end{array}$$

The dynamical system (3) is highly nonlinear, and hence, it is difficult to compute the endemic equilibrium point(s) explicitly in terms of model parameters; however, depending on the single infection model analyses, the complete dynamical system (3) endemic equilibrium *E*_*HC*_^∗^ = (*S*^∗^, *C*_*P*_^∗^, *H*_*P*_^∗^, *H*_*I*_^∗^, *C*_*I*_^∗^, *C*^∗^, *C*_*R*_^∗^, *H*_*T*_^∗^)  exists if  *ℛ*_*H*_ > 1 and *ℛ*_*C*_ > 1, i.e., *ℛ*_*HC*_^0^ > 1. We have discussed the complete model endemic equilibrium in the numerical analysis section.

#### 3.3.3. Analysis for the Possibility of Backward Bifurcation of the System (3)

Assume  *S* = *z*_1_, *C*_*P*_ = *z*_2_, *H*_*P*_ = *z*_3_,  *H*_*I*_ = *z*_4_,  *C*_*I*_ = *z*_5_,  *C* = *z*_6_,  *C*_*R*_ = *z*_7_, and  *H*_*I*_ = *z*_8_ such that *N* = *z*_1_ + *z*_2_ + *z*_3_ + *z*_4_ + *z*_5_ + *z*_6_ + *z*_7_ + *z*_8_.

Moreover, the vector representation  *Z* = (*z*_1_, *z*_2_, *z*_3_, *z*_4_, *z*_5_, *z*_6_, *z*_7_, *z*_8_)^*T*^, the dynamical system (3) is written as *dZ*/*dt* = *F*(*Z*) with *F* = (*f*_1_, *f*_2_, *f*_3_, *f*_4_, *f*_5_, *f*_6_, *f*_7_, *f*_8_)^*T*^, as

(37) $$\begin{array}{c} \frac{{dz}_{1}}{dt}=f_{1}=\left(1-\gamma_{1}-\gamma_{2}\right)\Gamma +\delta_{1}z_{2}+\delta_{2}z_{3}+\eta z_{7}-\left(\lambda_{H}+\lambda_{C}+\mu \right)z_{1},\\ \frac{{dz}_{2}}{dt}=f_{2}=\gamma_{1}\Gamma -\left(\delta \lambda_{H}+\delta_{1}+\mu \right)z_{2},\\ \frac{{dz}_{3}}{dt}=f_{3}=\gamma_{2}\Gamma -\left(\delta_{2}+\mu +\sigma \lambda_{C}\right)\delta_{3},\\ \frac{{dz}_{4}}{dt}=f=\lambda_{H}z_{1}+\delta \lambda_{H}z_{2}-\left(\mu +\mu_{1}+\gamma +\phi \lambda_{C}\right)z_{4},\\ \frac{{dz}_{5}}{dt}=f_{5}=\lambda_{C}z_{1}+\sigma \lambda_{C}z_{3}-\left(\kappa +\mu +\mu_{2}+\varphi \lambda_{H}\right)z_{5},\\ \frac{{dz}_{6}}{dt}=f_{6}=\varphi \lambda_{H}z_{5}+\phi \lambda_{C}z_{4}+\rho \lambda_{C}-\left(\mu +\mu_{3}+\theta \right)z_{6},\\ \frac{{dz}_{7}}{dt}=f_{7}=\kappa z_{5}-\left(\mu +\eta \right)z_{7},\\ \frac{{dz}_{8}}{dt}=f_{8}=\gamma z_{4}+\theta z_{6}-\rho \lambda_{C}-\mu z_{8}, \end{array}$$

with *λ*_*H*_ = *σ*_1_/*N*[*z*_4_ + *ρ*_1_*z*_6_] , 1 ≤ *ρ*_1_ < ∞,  *λ*_*C*_ = *σ*_2_/*N*[*z*_5_ + *ωz*_6_], and  1 ≤ *ω* < ∞. Then, the Jacobian matrix of the complete dynamical system (26) at  *E*_*HC*_^0^, represented by *J*(*E*_*HC*_^0^), is derived as

(38) $$\begin{array}{c} J\left(E_{HC}^{0}\right)=\left(\begin{array}{cccccccc} -\mu & \;\delta_{1} & \;\delta_{2} & \;F_{1} & F_{2} & F_{3} & \eta & 0\\ 0 & -\left(\delta_{1}+\mu \right) & 0 & \;F_{4} & 0 & F_{5} & 0 & 0\\ 0 & 0 & -\left(\delta_{2}+\mu \right) & 0 & F_{6} & F_{7} & 0 & 0\\ 0 & 0 & 0 & F_{8} & 0 & F_{9} & 0 & 0\\ 0 & 0 & 0 & 0 & F_{10} & F_{11} & 0 & \;0\\ 0 & 0 & 0 & 0 & 0 & -\left(\mu +\mu_{3}+\theta \right) & 0 & 0\\ 0 & 0 & 0 & 0 & \kappa & 0 & -\left(\mu +\eta \right) & 0\\ 0 & 0 & 0 & \gamma & 0 & \theta & 0 & -\mu \end{array}\right), \end{array}$$

where  *F*_1_ = −(*σ*_1_/*N*^0^)*z*_1_^0^,  *F*_2_ = −*σ*_2_*z*_1_^0^, *F*_3_ = −(*σ*_1_/*N*^0^)*ρ*_1_*z*_1_^0^ − *σ*_2_*ωz*_1_^0^,  *F*_4_ = −(*σ*_1_/*N*^0^)*z*_2_^0^, *F*_5_ = −(*σ*_1_/*N*^0^)*ρ*_1_*z*_2_^0^, *F*_6_ = −*σ*_2_*z*_3_^0^, *F*_7_ = −*σ*_2_*ωz*_3_^0^,  *F*_8_ = (*σ*_1_/*N*^0^)*z*_1_^0^ + (*σ*_1_/*N*^0^)*z*_2_^0^ − (*μ* + *μ*_1_ + *γ*), *F*_9_ = (*σ*_1_/*N*^0^)*ρ*_1_*z*_1_^0^ + (*σ*_1_/*N*^0^)*ρ*_1_*z*_2_^0^, *F*_10_ = *σ*_2_*z*_1_^0^ + *σ*_2_*z*_3_^0^ − (*κ* + *μ* + *μ*_2_), and *F*_11_ = *σ*_2_*ωz*_1_^0^ + *σ*_2_*ωz*_3_^0^.

Let us consider the case at *ℛ*_*C*_ > *ℛ*_*H*_ and *ℛ*_*HC*_^0^ = 1, so that *ℛ*_*C*_ = 1. Moreover, assume *σ*_2_ = *σ*^∗^ and taken as a bifurcation parameter. Calculating the expression for *σ*_2_ using *ℛ*_*C*_ = 1, i.e., *ℛ*_*C*_ = (*σ*_2_(*μ*(1 − *γ*_1_) + *δ*_1_))/((*μ* + *μ*_2_ + *κ*)(*μ* + *δ*_1_)) = 1, we computed the value *σ*^∗^ = *σ*_2_ = ((*μ* + *μ*_2_ + *κ*)(*μ* + *δ*_1_))/((*μ*(1 − *γ*_1_) + *δ*_1_)).

The eigenvalues of the matrix *J*(*E*_*HC*_^0^) of the dynamical system (26) at the DFE, with *σ*_2_ = *σ*^∗^, are calculated as

(39) $$\begin{array}{c} \zeta_{1}=-\mu <0\text{ or }\zeta_{2}=-\left(\delta_{1}+\mu \right)<0\text{ or }\zeta_{3}=-\left(\delta_{2}+\mu \right)<0\text{ or }\zeta_{4}=F_{8}=\frac{\sigma_{1}}{N^{0}}z_{1}^{0}+\frac{\delta_{1}}{N^{0}}z_{2}^{0}-\left(\mu +\mu_{1}+\gamma \right)=\left(\mu +\mu_{1}+\gamma \right)\left[R_{H}-1\right]<0\text{ whenever }R_{H}<1\text{ or }\zeta_{5}=0\text{ or }\zeta_{6}=-\left(\mu +\mu_{3}+\theta \right)<0\text{ or }\zeta_{7}=-\left(\mu +\eta \right)<0\text{ or }\zeta_{8}=-\mu <0. \end{array}$$

Therefore, every eigenvalue is negative if *ℛ*_*HC*_^0^ < 1 and also the matrix *J*(*E*_*HC*_^0^) of the system (26) at DFE, and  *σ*_2_ = *σ*^∗^, represented by *J*_*β*^∗^_, has a single zero eigenvalue (where every other eigenvalue has negative real part). Applying the Castillo-Chavez and Song criteria stated in [33] can be used to prove that the dynamical system (3) exhibits the phenomenon of forward bifurcation at  *ℛ*_*C*_ = 1. In the right and left eigenvectors of *J*_*β*^∗^_, at the case whenever *ℛ*_*C*_ = 1, the right eigenvector of the Jacobian of the dynamical system (37) at *σ*_2_ = *σ*^∗^ (represented by *J*_*β*^∗^_) corresponding to a simple zero eigenvalue is represented by *u* = (*y*_1_, *y*_2_, *y*_3_, *y*_4_, *y*_5_, *y*_6_, *y*_7_, *y*_8_)^*T*^

(40) $$\begin{array}{c} y_{1}=\frac{\delta_{2}F_{6}\left(\mu +\eta \right)y_{5}+\left(\delta_{2}+\mu \right)\left(\mu +\eta \right)F_{2}y_{5}+\left(\delta_{2}+\mu \right)\eta \kappa y_{5}}{\mu \left(\delta_{2}+\mu \right)\left(\mu +\eta \right)},\\ y_{2}=0,\\ y_{3}=\frac{F_{6}}{\delta_{2}+\mu }y_{5},\\ \;y_{4}=0,\\ y_{5}=y_{5}>0,\\ y_{6}=0,\\ y_{7}=\frac{\kappa }{\mu +\eta }y_{5},\\ y_{8}=0. \end{array}$$

Left eigenvectors corresponding to the simple zero eigenvalue at  *σ*_2_ = *σ*_2_^∗^ qualifying the product  *y*.*w* = 1, given as *w* = (*w*_1_, *w*_2_, *w*_3_, *w*_4_, *w*_5_, *w*_6_, *w*_7_, *w*_8_), are *w*_1_ = *w*_2_ = *w*_3_ = *w*_4_ = *w*_6_ = *w*_7_ = *w*_8_ = 0 and *w*_5_ = *w*_5_ > 0.

Using many steps of calculations, we have derived the bifurcation coefficients *a* and *b* given by

(41) $$\begin{array}{c} a=2w_{5}y_{1}y_{5}\frac{\partial^{2}f_{5}\left(0,0\right)}{\partial z_{1}\partial z_{5}}+2w_{5}y_{3}y_{5}\frac{\partial^{2}f_{5}\left(0,0\right)}{\partial z_{2}\partial z_{5}}=2\sigma_{2}^{*}w_{5}y_{5}\left[y_{1}+y_{3}\right],=2\sigma_{2}^{*}w_{5}y_{5}^{2}\left[\frac{-\delta_{2}\sigma_{2}y_{3}^{0}\left(\mu +\eta \right)-\left(\delta_{2}+\mu \right)\left(\mu +\eta \right)\sigma_{2}z_{1}^{0}-\left(\delta_{2}+\mu \right)\eta \kappa -\mu \left(\mu +\eta \right)\sigma_{2}z_{3}^{0}}{\mu \left(\delta_{2}+\mu \right)\left(\mu +\eta \right)}\right]. \end{array}$$

Then,

(42) $$\begin{array}{c} a=-2\sigma_{2}^{*}w_{5}y_{5}^{2}\left[\frac{\delta_{2}\sigma_{2}z_{3}^{0}\left(\mu +\eta \right)+\left(\delta_{2}+\mu \right)\left(\mu +\eta \right)\sigma_{2}z_{1}^{0}+\left(\delta_{2}+\mu \right)\eta \kappa +\mu \left(\mu +\eta \right)\sigma_{2}z_{3}^{0}}{\mu \left(\alpha_{2}+\mu \right)\left(\mu +\eta \right)}\right]<0,\\ b=w_{5}y_{5}\frac{\partial^{2}f_{5}\left(0,0\right)}{\partial z_{5}\partial \sigma_{2}}=w_{5}y_{5}\left(z_{3}^{0}+z_{1}^{0}\right)>0. \end{array}$$

Therefore, applying the Castillo-Chavez and Song criteria stated in [33] we have proved that the complete dynamical system (3) did not exhibit the phenomenon of backward bifurcation when  *ℛ*_*HC*_^0^ = *ℛ*_C_ = 1. Hence, only the disease-free equilibrium point given by

(43) $$\begin{array}{c} E_{HC}^{0}=\left({\text{S}}^{0},C_{P}^{0},H_{P}^{0},H_{I}^{0},C_{I}^{0},,{\text{C}}^{0},C_{R}^{0},H_{T}^{0}\right)=\left.\frac{\left(1-\gamma_{1}-\gamma_{2}\right)\Gamma \left(\delta_{1}+\mu \right)\left(\delta_{2}+\mu \right)+\delta_{1}\gamma_{1}\Gamma +\delta_{2}\gamma_{2}\Gamma \left(\delta_{1}+\mu \right)}{\mu \left(\delta_{1}+\mu \right)\left(\delta_{2}+\mu \right)},\frac{\gamma_{1}\Gamma }{\delta_{1}+\mu },\frac{\gamma_{2}\Gamma }{\delta_{2}+\mu },0,0,0,0,0\right) \end{array}$$

for the dynamical system (3) exists that means there is only DFE but not positive endemic equilibrium point in the region provided *ℛ*_*HC*_^0^ < 1.

Note: in the subsections represented by 3.1.1 and 3.2.1, we proved that DFE of the HBV and COVID-19 single infection models has global asymptotic stability when the associated effective reproduction number is less than one. Therefore, depending on the result and equation (42) the COVID-19 and HBV coinfection dynamical system (3) has a global asymptotic stability whenever  *ℛ*_*HC*_^0^ = max{*ℛ*_*H*_, *ℛ*_*C*_} < 1.

## 4. Numerical Simulation and Sensitivity Analysis

To verify the mathematical analysis results shown in the previous sections and subsections, we have carried out various sensitivity and numerical analyses. For the sensitivity and numerical analysis computations, we used parameter values adopting from different scholar studies and given the collection in Table 3.

### 4.1. Sensitivity Analysis Results

Definition: the variable *y* normalized forward sensitivity index which depends on a differentiable parameter *ξ* is defined by SI(*ϑ*) = (*∂y*/*∂ϑ*)∗(*ϑ*/*y*) [35, 36, 41, 55].

The sensitivity analysis is used to examine the most influential parameters in the spreading of the coinfection of HBV and COVID-19. From results of sensitivity analysis among others, the one which has a larger sensitivity index in magnitude is known as the most sensitive parameter. For this study, the sensitivity indices can be computed using the model effective reproduction numbers given by *ℛ*_*H*_ and *ℛ*_*C*_ since *ℛ*_*HC*_^0^ = max{*ℛ*_*H*_, *ℛ*_*C*_}.

Applying Table 3 (baseline values) of the model parameters, we have prepared the sensitivity index tables as Tables 4 and 5, respectively.

Using Table 3 (baseline values) of the model parameters, we have calculated the value of HBV effective reproduction number *ℛ*_*H*_ = 1.82 which implies that HBV infection spreads throughout the population. Also, Table 4 (sensitivity indices) shows that the HBV spreading rate *σ*_1_ has major effect on the HBV effective reproduction number denoted by *ℛ*_*H*_.

In a similar manner, applying values of the model parameters stated in Table 3 we calculated the numerical value of COVID-19 effective reproduction number given by *ℛ*_*C*_ = 3.23  which implies that the COVID-19 single infection is persistent throughout the population. Also, the sensitivity analysis given in Table 5 (sensitivity indices) shows that COVID-19 transmission rate  *σ*_2_ is the most sensitive model parameter which has great impact on the COVID-19 transmission. Comparing sensitivity indices given in Tables 4 and 5, one can conclude that the HBV transmission rate *σ*_1_ and COVID-19 spreading rate  *σ*_2_ are the most influential model parameters in the disease transmission, and stakeholders shall concentrate to control the values of these parameters by considering the suitable intervention strategies.

Simulation represented in Figure 2 shows the model parameter sensitivity indices graphically. From Figure 2 we can see that the model parameters *σ*_1_ and *σ*_2_ are highly sensitive with respect to the HBV infection and COVID-19 infection submodel effective reproduction numbers, respectively. Also, one can conclude that portions of protections *γ*_1_ and  *γ*_2_ and COVID-19 treatment rate *κ* are more sensitive parameters and important to control the disease transmission in the community.

### 4.2. Numerical Simulations

In this subsection, we carried out numerical analysis of the dynamical system (3). For simulations of the coinfection model (3) with nonnegative initial, we have used MATLAB ode45 with the embedded Runge-Kutta forward and backward numerical methods. In this part, we have investigated the model (3) endemic equilibrium point stability and the impacts of some basic model parameters on the model effective reproduction numbers and examined the effects of the proposed intervention strategies in the model construction. In this subsection for the case of numerical simulations to be performed, we have assumed the positive initial data given

(44) $$\begin{array}{c} \left(\text{S}\left(0\right),C_{P}\left(0\right),H_{P}\left(0\right),H_{I}\left(0\right),C_{I}\left(0\right),\text{C}\left(0\right),C_{R}\left(0\right),H_{T}\left(0\right)\right)=\left(1000,300,200,100,170,80,75,75\right), \end{array}$$

and used parameter baseline values given in Table 3.

#### 4.2.1. The Complete Model Simulation at *ℛ*_*HC*_^0^ < 1

In this subsection, we performed the complete coinfection model numerical simulation by considering the value of the model effective reproduction number as *ℛ*_*HC*_^0^max{*ℛ*_*H*_, *ℛ*_*C*_} = max{0.14, 0.26 } = 0.26 < 1, and the simulation result is illustrated in Figure 3. From Figure 3 we can observe that the simulation result justifies the analytical result, and after 20 days, the complete coinfection model (3) solutions will be converging to the disease-free equilibrium (DFE) point of the model.

#### 4.2.2. The Complete Model Simulation at *ℛ*_*HC*_^0^ > 1

In this subsection, we performed numerical simulation of the full dynamical system (3) using model parameter values given in Table 3 and we calculated for the value of the model effective reproduction number as *ℛ*_*HC*_^0^ = 3.23. The simulation result illustrated in Figure 4 shows that the model solutions are converging to the endemic equilibrium point of the model providing that *ℛ*_*HC*_^0^ = 3.23 > 1.

#### 4.2.3. Effect of HBV Transmission on COVID-19 Infection

Simulation illustrated in Figure 5 investigated to show the impact of HBV spreading rate *σ*_1_ on the number of HBV and COVID-19 coepidemic individuals *C*. From Figure 5 we observed that whenever the value of HBV spreading rate is going up, then the number of HBV and COVID-19 coinfectious individuals is going up throughout the population. Thus, increasing HBV spreading rate *σ*_1_ from 0.00001 to 0.8 leads to a highly increase of HBV and COVID-19 coepidemic number of individuals *C*.

#### 4.2.4. Impact of COVID-19 Spreads on HBV Infection

Numerical simulation given in Figure 6 investigated the impact of COVID-19 spreading rate *σ*_2_ on the number of HBV and COVID-19 coepidemic people *C*. From Figure 6 we observed that whenever the value of COVID-19 spreading rate *σ*_2_ increases, then the number of HBV and COVID-19 coinfectious individuals *C* is going up. Thus, increasing COVID-19 spreading rate *σ*_2_ from 0.00001 to 0.8 makes the HBV and COVID-19 coinfection *C* highly increases.

#### 4.2.5. Simulation to Investigate Effect of Treatment on HBV Infection

Numerical simulation shown in Figure 7 investigated the impact of HBV treatment on the HBV infectious individuals *H*_*I*_ throughout the community. From the result, we can conclude that when the value of treatment rate *γ* is going up, then the number of HBV infectious individuals *H*_*I*_ is going down. For the stakeholders, we recommend that they take their maximum effort to increase the value of HBV treatment rate to minimize the HBV transmission rate.

#### 4.2.6. Simulation to Investigate Effect of Treatment on Coinfection

In this subsection, numerical simulation represented in Figure 8 investigated the impact of COVID-19 treatment on the HBV and COVID-19 coinfectious individuals  *C*. From the result, we can conclude that whenever we increase the value of treatment rate *θ*, the number of coinfectious population is going down. Thus, whenever we increase the value of *θ* from 0.2 to 0.8, then the number of HBV and COVID-19 coinfectious individuals decreases through time.

#### 4.2.7. Simulation to Investigate the Effect of *σ*_1_ on *ℛ*_*H*_

Figure 9 depicts the HBV spreading rate *σ*_1_ highest direct impact on the HBV single infection model effective reproduction number *ℛ*_*H*_. From the numerical result, we observed that increasing the HBV spreading rate *σ*_1_ has a direct impact on its effective reproduction number  *ℛ*_*H*_. Thus, introducing protective and controlling strategies against HBV spreading is fundamental to minimized *σ*_1_ value less than 0.801.

#### 4.2.8. Simulation to Investigate the Effect of *γ*_2_ on *ℛ*_*H*_

Simulation illustrated in Figure 10 depicts that the recruitment rate portion *γ*_2_ has the highest indirect impact on the HBV submodel effective reproduction number *ℛ*_*H*_. The simulation result from Figure 10 shows whenever the value of *γ*_2_ increases then the HBV spreading rate decreases. Thus, applying the portion *γ*_2_ of the human recruitment rate Γ  to be more than 0.597 makes the value of *ℛ*_*H*_ less than one.

#### 4.2.9. Simulation to Investigate the Effect of *γ* on *ℛ*_*H*_

Figure 11 shows that the HBV treatment rate *γ* has influential indirect impact on *ℛ*_*H*_. We observed the result whenever we increase the treatment rate; then, the HBV transmission decreases in the community. Thus, applying the treatment rate *γ* to more than 0.898 made the value of the HBV infection effective reproduction number *ℛ*_*H*_ less than one.

#### 4.2.10. Simulation to Investigate the Effect of *σ*_2_ on *ℛ*_*C*_

Simulation illustrated in Figure 12 examined the effect of COVID-19 spreading rate *σ*_2_ on the COVID-19 subdynamical system (23) effective reproduction number *ℛ*_C_. From the figure, we observed that when the COVID-19 spreading rate value *σ*_2_ is going up implies the COVID-19 effective reproduction number increases, and whenever *σ*_2_ < 0.152 leads to *ℛ*_*C*_ < 1. Hence, we recommend for health stakeholders to give attention for minimizing the COVID-19 spreading rate *σ*_2_ to control and prevent COVID-19 transmission in the population. Epidemiologically, whenever the COVID-19 spreading rate increases, then the COVID-19 single infection is going up and the infection dies out from the community if *σ*_2_ < 0.152.

#### 4.2.11. Simulation to Investigate Impact of *γ*_1_ on *ℛ*_*C*_

Simulation given in Figure 13 depicts that a portion of COVID-19 protection *γ*_1_ has the highest indirect impact on the COVID-19 effective reproduction number *ℛ*_*C*_. We observed that whenever the value of *γ*_1_ increases, then the number of COVID-19 infectious population is going down throughout the community. Therefore, introducing a greater portion *γ*_1_ value than the value 0.898 made the value of the COVID-19 effective reproduction number *ℛ*_*C*_ below one.

#### 4.2.12. Simulation to Investigate Effect of *κ* on *ℛ*_*C*_

Numerical simulation represented in Figure 14 shows the indirect influence of the COVID-19 treatment rate (*κ*) on the COVID-19 effective reproduction number given by *ℛ*_*C*_. The result proved that whenever the COVID-19 treatment rate (*κ*) increases, then the value of *ℛ*_*C*_ is going down. As a result, giving the value of *κ* more than 0.758, then the value of *ℛ*_*C*_ is below one, and we recommend for the stakeholders to maximize the value of *κ*.

## 5. Conclusions

In this paper, we have constructed and investigated a continuous time dynamical model for the transmission of HBV and COVID-19 coinfection with protection and treatment strategies. The model incorporates three noninfectious groups, the susceptible group (*S*), the HBV protection group (*H*_*P*_), and the COVID-19 protection group (*C*_*P*_), and this made the model highly nonlinear and challenging for the qualitative analysis of the coinfection model. The model has been mathematically analyzed both for the submodels associating the cases that each disease type is isolated and in the case when there is HBV and COVID-19 coinfection. The proposed model includes the intervention strategies, protective as well as treatment, and numerical simulation of the deterministic model is presented. In the analysis, it has been indicated that the effect of protection as well as treating the infected ones with the available treatment mechanisms affects significantly the infection control strategy and its outcome. From the simulation results, it can be concluded that applying both protective and treatment control mechanisms simultaneously at the population level yields the most effective outcomes both economically and epidemiologically. Therefore, we strongly recommended to the stakeholders regarding economic as well as health issues to give more attention and the overall effort to implement both the protective and treatment control strategies simultaneously to minimize the HBV and COVID-19 single infections as well as the HBV and COVID-19 coinfection disease transmission in the community.

Any interested scholar can modify this study by considering the limitations of this study such as formulate a model which incorporate either of stochastic method, fractional order method, optimal control theory, age structure, or environmental effects, collect real data, and validate the formulated model.

## Figures and Tables

**Figure 1:** The flow chart of the coinfection of HBV and COVID-19 spreading dynamics with *λ*_*H*_(*t*) and *λ*_*C*_(*t*) given in (1) and (2), respectively.

**Figure 2:** Simulation of sensitivity indices of the model parameters with respect to *ℛ*_*HC*_^0^.

**Figure 3:** Convergence of the complete coinfection dynamics (3) solutions at *ℛ*_*HC*_^0^ = 0.26 < 1.

**Figure 4:** Convergence of the complete coinfection dynamics (3) solutions at *ℛ*_*HC*_^0^ = 3.23 > 1.

**Figure 5:** Impact of *σ*_1_ on *C*.

**Figure 6:** Impact of *σ*_2_ on *C*.

**Figure 7:** Impact of *γ* on *H*_*I*_.

**Figure 8:** Impact of *θ* on *C*.

**Figure 9:** Impact of *σ*_1_ on *ℛ*_*H*_.

**Figure 10:** Impact of *γ*_2_ on *ℛ*_*H*_.

**Figure 11:** Impact of *γ* on *ℛ*_*H*_.

**Figure 12:** Impact of *σ*_2_ on *ℛ*_*C*_.

**Figure 13:** Impact of *γ*_1_ on *ℛ*_*C*_.

**Figure 14:** Impact of *κ* on *ℛ*_*C*_.

**Table 1:** Definitions of the model parameters.

Parameter	Definition
*μ*_1_	HBV death rate
*μ*_2_	COVID-19-induced death rate
*μ*_3_	Death rate by HBV and COVID-19 coinfection
*δ*_1_	Protection lose rate of COVID-19
*δ*_2_	Protection lose rate of HBV
*σ*_1_	Spreading rate of HBV
*σ*_2_	Spreading rate of COVID-19
*γ*	HBV infection treatment rate
𝛿	Modification parameter
*η*	Immunity lose rate of COVID-19
*θ*	Treatment rate of the coinfected group
*κ*	Recovery rate of COVID-19
*μ*	Natural death rate
*σ*_1_	Portion entered to the COVID-19 protection group
*σ*_2_	Portion entered to the HBV protection group
*ρ*	Modification parameter
*σ*	Modification parameter
*φ*	Modification parameter
*Φ*	Modification parameter
Γ	Individual recruitment rate

**Table 2:** Interpretation of state variables.

Variable	Interpretation
*S*	Susceptible group
*C*_*P*_	COVID-19-protected group
*H*_*P*_	HBV-protected group
*H*_*I*_	HBV-infected group
*C*_*I*_	COVID-19-infected group
*C*	HBV and COVID-19 coinfected group
*C*_*R*_	COVID-19-recovered group
*H*_*T*_	HBV-treated group

**Table 3:** Values for parameters.

Parameter	Value	Source
*μ*_1_	0.0200/day	[3]
*μ*_2_	0.0214/day	[3]
*μ*_3_	0.0500/day	[3]
*δ*_1_	0.0015/day	Assumed
*δ*_2_	0.0004/day	Estimated [43]
*σ*_1_	5.0 × 10^−8^/day	[3]
*σ*_2_	6.29 × 10^−8^/day	[3]
*γ*	0.5/day	[3]
𝛿	1 no. unit	Assumed
*η*	0.002/day	Assumed
*θ*	0.15/day	[3]
*κ*	0.005/day	[28]
*μ*	(1/64.5^∗^365)/day	[14]
*γ*_1_	0.012/day	Assumed
*γ*_2_	0.5813/day	Assumed
*ρ*	1 no. unit	Assumed
*σ*	1 no. unit	Assumed
*φ*	1 no. unit	Assumed
*Φ*	1.2 no. unit	[14]
Δ	1000 humans/day	[28]

**Table 4:** Sensitivity indices of *ℛ*_*HC*_^0^ = *ℛ*_*H*_.

Sensitivity index	Values
SI(*σ*_1_)	+1
SI(*δ*_2_)	0.04
SI(*γ*_2_)	-0.68
SI(*μ*_1_)	0.390
SI(*γ*)	-0. 69

**Table 5:** Sensitivity indices of *ℛ*_*HC*_^0^ = *ℛ*_*C*_.

Sensitivity index	Value
SI(*σ*_2_)	+1
SI(*μ*_2_)	0.02
SI(*κ*)	-0.68
SI(*δ*_1_)	0.34
SI(*γ*_1_)	-0.67

## Data Availability

Data used to support the findings of this study are included in the article.
